RETRACTED

# *catena*-Poly[[aqua­(2,2′-bipyridyl)cobalt(II)]-μ-5-nitro­isophthalato]

**DOI:** 10.1107/S1600536808038178

**Published:** 2008-11-22

**Authors:** Ying Liu, Qingpeng He, Xianxi Zhang, Zechun Xue, Chunyan Lv

**Affiliations:** a College of Chemistry and Chemical Engineering, Liaocheng University, Liaocheng 252059, People’s Republic of China

## Abstract

In the crystal structure of the title compound, [Co(C_8_H_3_NO_6_)(C_10_H_8_N_2_)(H_2_O)]_*n*_, there are two symmetry-independent one-dimensional coordination polymers, which are approximately related by noncrystallographic inversion symmetry. Each zigzag chain is constructed from one Co^II^ ion, one *O*-monodentate 5-nitro­isophthalate (ndc) dianion, one *N*,*N*′-bidentate 2,2′-bipyridyl ligand and one water mol­ecule. A symmetry-generated *O*,*O*′-bidentate ndc dianion completes the cobalt coordination environment, which could be described as very distorted cis-CoN_2_O_4_ octa­hedral. The bridging ndc ligands result in parallel chains running along the *a* direction, and O—H⋯O hydrogen bonds arising from the water mol­ecules complete the structure.

## Related literature

For uses of carboxylic acids in materials science, see: Church & Halvorson (1959 ▶); and in biological systems, see: Okabe & Oya (2000 ▶).

## Experimental

### 

#### Crystal data

[Co(C_8_H_3_NO_6_)(C_10_H_8_N_2_)(H_2_O)]
*M* *_r_* = 442.24
Monoclinic,
*a* = 10.0125 (10) Å
*b* = 23.575 (2) Å
*c* = 15.403 (2) Å
β = 97.28 (1)°
*V* = 3606.3 (7) Å^3^
*Z* = 8
Mo *K*α radiation
μ = 1.00 mm^−1^
*T* = 293 (2) K
0.43 × 0.28 × 0.20 mm

#### Data collection

Bruker APEXII CCD diffractometer
Absorption correction: multi-scan (*SADABS*; Bruker, 2001 ▶) *T*_min_ = 0.673, *T*_max_ = 0.825
18893 measured reflections
6672 independent reflections
5103 reflections with *I* > 2σ(*I*)
*R*_int_ = 0.025

#### Refinement

*R*[*F* ^2^ > 2σ(*F* ^2^)] = 0.037
*wR*(*F* ^2^) = 0.106
*S* = 1.01
6672 reflections
535 parameters
6 restraints
H atoms treated by a mixture of independent and constrained refinement
Δρ_max_ = 0.95 e Å^−3^
Δρ_min_ = −0.29 e Å^−3^

### 

Data collection: *APEX2* (Bruker, 2004 ▶); cell refinement: *SAINT-Plus* (Bruker, 2001 ▶); data reduction: *SAINT-Plus*; program(s) used to solve structure: *SHELXS97* (Sheldrick, 2008 ▶); program(s) used to refine structure: *SHELXL97* (Sheldrick, 2008 ▶); molecular graphics: *SHELXTL* (Sheldrick, 2008 ▶); software used to prepare material for publication: *SHELXTL*.

## Supplementary Material

Crystal structure: contains datablocks global, I. DOI: 10.1107/S1600536808038178/hb2844sup1.cif

Structure factors: contains datablocks I. DOI: 10.1107/S1600536808038178/hb2844Isup2.hkl

Additional supplementary materials:  crystallographic information; 3D view; checkCIF report

RETRACTED

## Figures and Tables

**Table 1:** Selected bond lengths (Å)

Co1—N2	2.065 (2)
Co1—N1	2.075 (2)
Co1—O2	2.0369 (19)
Co1—O1*W*	2.102 (2)
Co1—O5^i^	2.131 (2)
Co1—O6^i^	2.257 (2)
Co2—N3	2.073 (2)
Co2—N4	2.078 (3)
Co2—O12	2.031 (2)
Co2—O2*W*	2.089 (2)
Co2—O10^ii^	2.116 (2)
Co2—O9^ii^	2.294 (2)

Symmetry codes: (i) ; (ii) .

**Table 2:** Hydrogen-bond geometry (Å, °)

*D*—H⋯*A*	*D*—H	H⋯*A*	*D*⋯*A*	*D*—H⋯*A*
O1*W*—H1*W*⋯O12^i^	0.830 (10)	2.01 (2)	2.771 (3)	153 (3)
O2*W*—H4*W*⋯O2^ii^	0.831 (10)	1.957 (17)	2.747 (3)	159 (3)
O1*W*—H2*W*⋯O9	0.830 (10)	2.05 (2)	2.763 (3)	143 (3)
O2*W*—H3*W*⋯O6	0.835 (10)	2.10 (3)	2.781 (3)	138 (3)

Symmetry codes: (i) ; (ii) .

## supplementary crystallographic information

### Comment

In recent years, carboxylic acids have been widely used as polydentate ligands, which can coordinate to transition or rare earth ions yielding complexes with interesting properties that are useful in materials science (Church & Halvorson, 1959) and in biological systems (Okabe & Oya, 2000). The importance of transition metal dicarboxylate complexes motivated us to pursue synthetic strategies for these compounds, using 5-nitroisophthalic acid as a polydentate ligand. Here we report the synthesis and X-ray crystal structure analysis of the title compound, (I), (Fig. 1).

Compound (I) is constructed from two zigzag chains, each containing one Co^II^ atom, one O-monodentate 5-nitroisophthalato (ndc) dianion, one N,N-bidentate 2,2'-bipyridyl ligand and one water molecule. A symmetry-generated, O,O-bidentate ndc dianion completes the cobalt coordination, which could be described as very distorted cis-CoN_2_O_4_ octahedral (Table 1). The bridging ndc ligands result in parallel chains running along the a direction (Fig. 2) and O—H···O hydrogen bonds arising from the water molecules (Table 2) complete the structure (Fig. 3).

### Experimental

A mixture of cobalt dichloride (0.5 mmol), 2,2'-bipyridine (0.5 mmol), and 5-nitroisophthalic acid (0.5 mmol) in H_2_O (8 ml) and ethanol (8 ml) sealed in a 25 ml Teflon-lined stainless steel autoclave was kept at 413 K for three days. Red blocks of (I) were obtained after cooling to room temperature with a yield of 27%. Anal. Calc. for C_18_H_13_CoN_3_O_7_: C 48.34, H 2.91, N 10.74%; Found: C 48.30, H 2.84, N 10.69%.

### Refinement

The H atoms of the water molecules were located from difference density maps and were refined with distance restraints of H···H = 1.38 (2) Å, O—H = 0.88 (2) Å, and with a fixed *U*_iso_ of 0.80 Å^2^. All other H atoms were placed in calculated positions with C—H = 0.93 Å and refined as riding with *U*_iso_(H) = 1.2*U*_eq_(carrier).

RETRACTED

### Crystal data

**Table:**

[Co(C_8_H_3_NO_6_)(C_10_H_8_N_2_)(H_2_O)]	*F*_000_ = 1800
*M**_r_* = 442.24	*D*_x_ = 1.629 Mg m^−^^3^
Monoclinic, *P*2_1_/*n*	Mo *K*α radiation λ = 0.71073 Å
Hall symbol: -P 2yn	Cell parameters from 6672 reflections
*a* = 10.0125 (10) Å	θ = 1.7–25.5º
*b* = 23.575 (2) Å	µ = 1.00 mm^−^^1^
*c* = 15.403 (2) Å	*T* = 293 (2) K
β = 97.28 (1)º	Block, red
*V* = 3606.3 (7) Å^3^	0.43 × 0.28 × 0.20 mm
*Z* = 8	

### Data collection

**Table:**

Bruker APEXII CCD diffractometer	6672 independent reflections
Radiation source: fine-focus sealed tube	5103 reflections with *I* > 2σ(*I*)
Monochromator: graphite	*R*_int_ = 0.025
*T* = 293(2) K	θ_max_ = 25.5º
ω scans	θ_min_ = 1.7º
Absorption correction: multi-scan(SADABS; Bruker, 2001)	*h* = −12→10
*T*_min_ = 0.673, *T*_max_ = 0.825	*k* = −28→22
18893 measured reflections	*l* = −18→18

### Refinement

**Table:**

Refinement on *F*^2^	Secondary atom site location: difference Fourier map
Least-squares matrix: full	Hydrogen site location: inferred from neighbouring sites
*R*[*F*^2^ > 2σ(*F*^2^)] = 0.037	H atoms treated by a mixture of independent and constrained refinement
*wR*(*F*^2^) = 0.106	*w* = 1/[σ^2^(*F*_o_^2^) + (0.0548*P*)^2^ + 2.8058*P*] where *P* = (*F*_o_^2^ + 2*F*_c_^2^)/3
*S* = 1.01	(Δ/σ)_max_ = 0.032
6672 reflections	Δρ_max_ = 0.95 e Å^−^^3^
535 parameters	Δρ_min_ = −0.29 e Å^−^^3^
6 restraints	Extinction correction: none
Primary atom site location: structure-invariant direct methods	

### Special details

**Table:**

Geometry. All e.s.d.'s (except the e.s.d. in the dihedral angle between two l.s. planes) are estimated using the full covariance matrix. The cell e.s.d.'s are taken into account individually in the estimation of e.s.d.'s in distances, angles and torsion angles; correlations between e.s.d.'s in cell parameters are only used when they are defined by crystal symmetry. An approximate (isotropic) treatment of cell e.s.d.'s is used for estimating e.s.d.'s involving l.s. planes.
Refinement. Refinement of *F*^2^ against ALL reflections. The weighted *R*-factor *wR* and goodness of fit *S* are based on *F*^2^, conventional *R*-factors *R* are based on *F*, with *F* set to zero for negative *F*^2^. The threshold expression of *F*^2^ > σ(*F*^2^) is used only for calculating *R*-factors(gt) *etc*. and is not relevant to the choice of reflections for refinement. *R*-factors based on *F*^2^ are statistically about twice as large as those based on *F*, and *R*- factors based on ALL data will be even larger.

### Fractional atomic coordinates and isotropic or equivalent isotropic displacement parameters (Å^2^)

**Table:**

	*x*	*y*	*z*	*U*_iso_*/*U*_eq_	
Co1	1.16169 (4)	0.154445 (14)	0.85573 (2)	0.02466 (11)	
Co2	0.12374 (4)	0.354444 (15)	0.93350 (3)	0.02797 (12)	
C1	0.0858 (3)	0.43912 (15)	0.7845 (2)	0.0469 (8)	
H1	0.0715	0.4073	0.7489	0.056*	
C2	0.0708 (4)	0.49272 (17)	0.7466 (3)	0.0555 (10)	
H2	0.0482	0.4963	0.6864	0.067*	
C3	0.0893 (4)	0.54031 (16)	0.7979 (3)	0.0570 (10)	
H3	0.0810	0.5763	0.7731	0.068*	
C4	0.1204 (3)	0.53368 (14)	0.8864 (3)	0.0474 (9)	
H4	0.1307	0.5651	0.9231	0.057*	
C5	0.1365 (3)	0.47893 (12)	0.9205 (2)	0.0363 (7)	
C6	0.1704 (3)	0.46688 (12)	1.0143 (2)	0.0361 (7)	
C7	0.1997 (3)	0.50925 (14)	1.0774 (3)	0.0490 (9)	
H7	0.1978	0.5474	1.0616	0.059*	
C8	0.2313 (3)	0.49307 (17)	1.1631 (3)	0.0557 (10)	
H8	0.2506	0.5203	1.2067	0.067*	
C9	0.2341 (4)	0.43613 (17)	1.1843 (3)	0.0559 (10)	
H9	0.2569	0.4248	1.2421	0.067*	
C10	0.2034 (3)	0.39623 (15)	1.1200 (2)	0.0468 (8)	
H10	0.2049	0.3580	1.1351	0.056*	
C11	0.5280 (3)	0.24937 (12)	1.02748 (19)	0.0320 (6)	
H11	0.4449	0.2352	1.0380	0.038*	
C12	0.6449 (3)	0.22104 (12)	1.05893 (19)	0.0321 (6)	
C13	0.7703 (3)	0.24074 (12)	1.04616 (19)	0.0327 (7)	
H13	0.8479	0.2213	1.0685	0.039*	
C14	0.7776 (3)	0.29080 (11)	0.99863 (18)	0.0271 (6)	
C15	0.9110 (3)	0.31378 (12)	0.9803 (2)	0.0312 (6)	
C16	0.6606 (3)	0.31947 (12)	0.96577 (18)	0.0286 (6)	
H16	0.6666	0.3527	0.9339	0.034*	
C17	0.5354 (3)	0.29914 (12)	0.98002 (18)	0.0288 (6)	
C18	0.4121 (3)	0.33266 (13)	0.9446 (2)	0.0325 (7)	
C19	1.1953 (4)	0.07221 (15)	1.0079 (2)	0.0512 (9)	
H19	1.2137	0.1044	1.0424	0.061*	
C20	1.2036 (5)	0.01944 (18)	1.0474 (3)	0.0684 (12)	
H20	1.2268	0.0164	1.1076	0.082*	
C21	1.1774 (5)	−0.02879 (17)	0.9971 (3)	0.0688 (12)	
H21	1.1813	−0.0645	1.0230	0.083*	
C22	1.1455 (4)	−0.02303 (14)	0.9087 (2)	0.0526 (9)	
H22	1.1289	−0.0547	0.8731	0.063*	
C23	1.1386 (3)	0.03108 (12)	0.8732 (2)	0.0327 (7)	
C24	1.1073 (3)	0.04138 (12)	0.7783 (2)	0.0314 (6)	
C25	1.0794 (3)	−0.00192 (13)	0.7180 (2)	0.0411 (8)	
H25	1.0787	−0.0396	0.7357	0.049*	
C26	1.0526 (3)	0.01263 (15)	0.6307 (2)	0.0456 (8)	
H26	1.0329	−0.0152	0.5883	0.055*	
C27	1.0556 (3)	0.06936 (15)	0.6071 (2)	0.0459 (8)	
H27	1.0365	0.0798	0.5486	0.055*	
C28	1.0866 (3)	0.11017 (13)	0.6701 (2)	0.0381 (7)	
H28	1.0889	0.1480	0.6532	0.046*	
C29	0.8750 (3)	0.17566 (13)	0.8380 (2)	0.0336 (7)	
C30	0.7500 (3)	0.20949 (12)	0.80607 (18)	0.0274 (6)	
C31	0.7569 (3)	0.26263 (12)	0.76643 (19)	0.0314 (6)	
H31	0.8396	0.2780	0.7575	0.038*	
C32	0.6258 (3)	0.18764 (12)	0.81981 (19)	0.0297 (6)	
H32	0.6210	0.1529	0.8477	0.036*	
C33	0.6392 (3)	0.29172 (12)	0.7409 (2)	0.0347 (7)	
C34	0.5084 (3)	0.21757 (12)	0.79203 (18)	0.0273 (6)	
C35	0.5143 (3)	0.27061 (13)	0.75206 (19)	0.0332 (7)	
H35	0.4363	0.2910	0.7336	0.040*	
C36	0.3756 (3)	0.19401 (13)	0.8104 (2)	0.0331 (7)	
H1W	1.243 (3)	0.2304 (11)	0.958 (3)	0.080*	
H2W	1.126 (2)	0.2153 (14)	0.989 (3)	0.080*	
H3W	0.164 (2)	0.2956 (15)	0.803 (3)	0.080*	
H4W	0.042 (3)	0.2778 (10)	0.823 (3)	0.080*	
N1	1.1134 (2)	0.09709 (10)	0.75443 (15)	0.0302 (5)	
N2	1.1617 (3)	0.07823 (10)	0.92182 (16)	0.0349 (6)	
N3	0.1199 (2)	0.43207 (10)	0.87001 (17)	0.0349 (6)	
N4	0.1713 (2)	0.41090 (10)	1.03641 (17)	0.0361 (6)	
N5	0.6352 (3)	0.16753 (12)	1.10790 (19)	0.0477 (7)	
N6	0.6479 (3)	0.34937 (13)	0.7036 (2)	0.0578 (9)	
O1	0.8634 (2)	0.12806 (12)	0.8691 (2)	0.0705 (9)	
O2	0.98644 (19)	0.19824 (8)	0.82627 (15)	0.0379 (5)	
O3	0.7556 (3)	0.37273 (12)	0.7088 (2)	0.0801 (10)	
O4	0.5459 (3)	0.37066 (17)	0.6681 (3)	0.1342 (19)	
O5	0.3733 (2)	0.14822 (9)	0.85254 (16)	0.0440 (6)	
O6	0.26919 (19)	0.22039 (9)	0.78407 (15)	0.0422 (5)	
O7	0.5264 (3)	0.14506 (14)	1.1063 (2)	0.0932 (12)	
O8	0.7366 (3)	0.14819 (11)	1.14856 (19)	0.0642 (8)	
O9	1.0167 (2)	0.28717 (9)	1.00726 (15)	0.0411 (5)	
O10	0.9137 (2)	0.35927 (9)	0.93795 (16)	0.0442 (6)	
O11	0.4241 (2)	0.37689 (11)	0.90426 (18)	0.0586 (7)	
O12	0.30031 (19)	0.31194 (9)	0.96161 (15)	0.0409 (5)	
O1W	1.1948 (2)	0.20370 (8)	0.97017 (15)	0.0371 (5)	
O2W	0.0917 (2)	0.30554 (8)	0.81966 (16)	0.0374 (5)	

RETRACTED

### Atomic displacement parameters (Å^2^)

**Table:**

	*U*^11^	*U*^22^	*U*^33^	*U*^12^	*U*^13^	*U*^23^
Co1	0.01864 (19)	0.02268 (19)	0.0325 (2)	0.00142 (14)	0.00270 (15)	0.00151 (15)
Co2	0.01822 (19)	0.0237 (2)	0.0425 (2)	0.00121 (14)	0.00602 (16)	0.00113 (16)
C1	0.0428 (19)	0.048 (2)	0.052 (2)	0.0030 (15)	0.0148 (16)	0.0066 (16)
C2	0.046 (2)	0.065 (3)	0.057 (2)	0.0082 (18)	0.0139 (18)	0.024 (2)
C3	0.043 (2)	0.042 (2)	0.090 (3)	0.0027 (16)	0.020 (2)	0.026 (2)
C4	0.0326 (18)	0.0322 (17)	0.080 (3)	0.0017 (14)	0.0173 (17)	0.0057 (17)
C5	0.0193 (14)	0.0299 (15)	0.062 (2)	−0.0004 (12)	0.0141 (14)	0.0001 (14)
C6	0.0188 (14)	0.0342 (16)	0.057 (2)	−0.0007 (12)	0.0101 (13)	−0.0045 (14)
C7	0.0352 (18)	0.0352 (18)	0.078 (3)	−0.0024 (14)	0.0127 (18)	−0.0098 (17)
C8	0.038 (2)	0.067 (3)	0.062 (3)	−0.0018 (17)	0.0042 (18)	−0.022 (2)
C9	0.043 (2)	0.073 (3)	0.052 (2)	0.0057 (18)	0.0078 (17)	−0.0072 (19)
C10	0.0398 (19)	0.051 (2)	0.050 (2)	0.0067 (16)	0.0065 (16)	0.0001 (17)
C11	0.0204 (14)	0.0411 (16)	0.0348 (17)	−0.0058 (12)	0.0051 (12)	0.0010 (13)
C12	0.0267 (15)	0.0373 (16)	0.0323 (16)	−0.0020 (12)	0.0039 (12)	0.0048 (12)
C13	0.0210 (14)	0.0419 (17)	0.0347 (17)	0.0023 (12)	0.0012 (12)	0.0005 (13)
C14	0.0194 (14)	0.0317 (14)	0.0313 (15)	−0.0005 (11)	0.0069 (11)	−0.0043 (12)
C15	0.0185 (14)	0.0359 (16)	0.0403 (17)	0.0013 (12)	0.0077 (12)	−0.0087 (13)
C16	0.0228 (14)	0.0299 (14)	0.0336 (16)	−0.0011 (11)	0.0054 (12)	−0.0007 (12)
C17	0.0194 (14)	0.0358 (16)	0.0310 (16)	0.0001 (11)	0.0023 (11)	−0.0047 (12)
C18	0.0209 (15)	0.0387 (17)	0.0373 (17)	0.0023 (12)	0.0010 (12)	−0.0054 (13)
C19	0.070 (3)	0.048 (2)	0.0355 (19)	0.0013 (18)	0.0076 (17)	0.0048 (15)
C20	0.102 (4)	0.065 (3)	0.038 (2)	0.005 (2)	0.009 (2)	0.0146 (19)
C21	0.096 (3)	0.046 (2)	0.063 (3)	0.002 (2)	0.008 (2)	0.030 (2)
C22	0.068 (3)	0.0338 (18)	0.056 (2)	−0.0038 (17)	0.0053 (19)	0.0100 (16)
C23	0.0258 (15)	0.0308 (15)	0.0415 (18)	−0.0007 (12)	0.0043 (12)	0.0044 (13)
C24	0.0230 (14)	0.0304 (15)	0.0408 (17)	−0.0015 (12)	0.0042 (12)	0.0016 (13)
C25	0.0343 (17)	0.0329 (16)	0.056 (2)	−0.0028 (13)	0.0052 (15)	−0.0044 (15)
C26	0.0389 (19)	0.051 (2)	0.046 (2)	−0.0031 (15)	0.0035 (15)	−0.0147 (16)
C27	0.045 (2)	0.055 (2)	0.0367 (18)	0.0019 (16)	−0.0003 (15)	−0.0041 (15)
C28	0.0405 (18)	0.0378 (17)	0.0353 (17)	0.0061 (14)	0.0027 (14)	0.0054 (13)
C29	0.0221 (15)	0.0413 (17)	0.0369 (17)	0.0018 (13)	0.0017 (12)	0.0045 (13)
C30	0.0185 (14)	0.0351 (15)	0.0285 (15)	0.0014 (11)	0.0021 (11)	−0.0006 (12)
C31	0.0192 (14)	0.0402 (16)	0.0351 (16)	−0.0014 (12)	0.0045 (12)	0.0051 (13)
C32	0.0256 (15)	0.0311 (15)	0.0328 (15)	−0.0014 (12)	0.0060 (12)	−0.0004 (12)
C33	0.0303 (16)	0.0368 (16)	0.0379 (17)	0.0033 (13)	0.0078 (13)	0.0108 (13)
C34	0.0193 (13)	0.0346 (15)	0.0284 (15)	−0.0007 (11)	0.0047 (11)	−0.0063 (12)
C35	0.0215 (14)	0.0439 (17)	0.0340 (16)	0.0086 (12)	0.0030 (12)	0.0023 (13)
C36	0.0240 (15)	0.0401 (17)	0.0361 (17)	−0.0022 (13)	0.0070 (12)	−0.0110 (13)
N1	0.0251 (12)	0.0298 (12)	0.0358 (14)	0.0034 (10)	0.0039 (10)	0.0004 (10)
N2	0.0335 (14)	0.0349 (14)	0.0369 (15)	−0.0008 (11)	0.0067 (11)	0.0042 (11)
N3	0.0247 (13)	0.0352 (14)	0.0458 (17)	0.0018 (10)	0.0085 (11)	0.0055 (11)
N4	0.0264 (13)	0.0343 (14)	0.0483 (16)	0.0041 (10)	0.0079 (11)	−0.0007 (11)
N5	0.0348 (16)	0.0546 (17)	0.0532 (18)	−0.0040 (14)	0.0034 (13)	0.0203 (14)
N6	0.0458 (19)	0.0573 (19)	0.073 (2)	0.0145 (16)	0.0191 (16)	0.0331 (16)
O1	0.0359 (14)	0.0722 (18)	0.105 (2)	0.0136 (13)	0.0152 (14)	0.0578 (17)
O2	0.0161 (10)	0.0346 (11)	0.0623 (14)	0.0004 (8)	0.0022 (9)	−0.0024 (10)
O3	0.065 (2)	0.0644 (18)	0.108 (2)	−0.0176 (15)	−0.0012 (17)	0.0410 (17)
O4	0.0504 (19)	0.129 (3)	0.228 (5)	0.039 (2)	0.036 (2)	0.134 (3)
O5	0.0274 (12)	0.0441 (13)	0.0621 (15)	−0.0034 (9)	0.0117 (10)	0.0051 (11)
O6	0.0187 (10)	0.0491 (13)	0.0594 (15)	0.0039 (9)	0.0073 (10)	−0.0021 (11)
O7	0.0504 (18)	0.100 (2)	0.123 (3)	−0.0321 (16)	−0.0136 (18)	0.068 (2)
O8	0.0439 (15)	0.0619 (17)	0.087 (2)	0.0111 (12)	0.0070 (14)	0.0357 (14)
O9	0.0185 (10)	0.0453 (12)	0.0603 (14)	0.0035 (9)	0.0079 (10)	−0.0007 (10)
O10	0.0276 (11)	0.0363 (12)	0.0711 (16)	−0.0028 (9)	0.0161 (11)	0.0094 (11)
O11	0.0374 (14)	0.0576 (16)	0.0799 (18)	0.0077 (11)	0.0040 (13)	0.0303 (14)
O12	0.0190 (10)	0.0378 (12)	0.0658 (15)	0.0009 (9)	0.0052 (10)	−0.0032 (10)
O1W	0.0303 (12)	0.0335 (11)	0.0465 (13)	0.0030 (9)	0.0009 (10)	−0.0036 (9)
O2W	0.0287 (11)	0.0335 (11)	0.0502 (13)	0.0025 (9)	0.0050 (10)	0.0004 (10)

RETRACTED

### Geometric parameters (Å, °)

**Table:**

Co1—N2	2.065 (2)	C19—C20	1.382 (5)
Co1—N1	2.075 (2)	C19—H19	0.9300
Co1—O2	2.0369 (19)	C20—C21	1.382 (6)
Co1—O1W	2.102 (2)	C20—H20	0.9300
Co1—O5^i^	2.131 (2)	C21—C22	1.365 (5)
Co1—O6^i^	2.257 (2)	C21—H21	0.9300
Co2—N3	2.073 (2)	C22—C23	1.386 (4)
Co2—N4	2.078 (3)	C22—H22	0.9300
Co2—O12	2.031 (2)	C23—N2	1.344 (4)
Co2—O2W	2.089 (2)	C23—C24	1.475 (4)
Co2—O10^ii^	2.116 (2)	C24—N1	1.367 (4)
Co2—O9^ii^	2.294 (2)	C24—C25	1.385 (4)
C1—N3	1.329 (4)	C25—C26	1.380 (5)
C1—C2	1.392 (5)	C25—H25	0.9300
C1—H1	0.9300	C26—C27	1.387 (5)
C2—C3	1.372 (6)	C26—H26	0.9300
C2—H2	0.9300	C27—C28	1.374 (4)
C3—C4	1.367 (6)	C27—H27	0.9300
C3—H3	0.9300	C28—N1	1.329 (4)
C4—C5	1.395 (4)	C28—H28	0.9300
C4—H4	0.9300	C29—O1	1.231 (4)
C5—N3	1.349 (4)	C29—O2	1.270 (3)
C5—C6	1.470 (5)	C29—C30	1.513 (4)
C6—N4	1.362 (4)	C30—C32	1.386 (4)
C6—C7	1.398 (5)	C30—C31	1.399 (4)
C7—C8	1.373 (5)	C31—C33	1.377 (4)
C7—H7	0.9300	C31—H31	0.9300
C8—C9	1.381 (5)	C32—C34	1.391 (4)
C8—H8	0.9300	C32—H32	0.9300
C9—C10	1.372 (5)	C33—C35	1.377 (4)
C9—H9	0.9300	C33—N6	1.482 (4)
C10—N4	1.332 (4)	C34—C35	1.398 (4)
C10—H10	0.9300	C34—C36	1.500 (4)
C11—C12	1.381 (4)	C35—H35	0.9300
C11—C17	1.389 (4)	C36—O6	1.256 (3)
C11—H11	0.9300	C36—O5	1.261 (4)
C12—C13	1.376 (4)	C36—Co1^ii^	2.515 (3)
C12—N5	1.479 (4)	N5—O7	1.209 (4)
C13—C14	1.396 (4)	N5—O8	1.212 (3)
C13—H13	0.9300	N6—O3	1.204 (4)
C14—C16	1.390 (4)	N6—O4	1.205 (4)
C14—C15	1.501 (4)	O5—Co1^ii^	2.131 (2)
C15—O9	1.255 (3)	O6—Co1^ii^	2.257 (2)
C15—O10	1.257 (4)	O9—Co2^i^	2.294 (2)
C16—C17	1.386 (4)	O10—Co2^i^	2.116 (2)
C16—H16	0.9300	O1W—H1W	0.830 (10)
C17—C18	1.508 (4)	O1W—H2W	0.830 (10)
C18—O11	1.228 (4)	O2W—H3W	0.835 (10)
C18—O12	1.278 (3)	O2W—H4W	0.831 (10)
C19—N2	1.334 (4)		
			
O2—Co1—N2	119.80 (9)	C20—C19—H19	119.1
O2—Co1—N1	92.92 (9)	C19—C20—C21	119.9 (4)
N2—Co1—N1	77.83 (9)	C19—C20—H20	120.1
O2—Co1—O1W	86.94 (8)	C21—C20—H20	120.1
N2—Co1—O1W	94.42 (9)	C22—C21—C20	118.7 (3)
N1—Co1—O1W	171.00 (9)	C22—C21—H21	120.6
O2—Co1—O5^i^	149.41 (9)	C20—C21—H21	120.6
N2—Co1—O5^i^	90.78 (9)	C21—C22—C23	118.6 (3)
N1—Co1—O5^i^	94.31 (9)	C21—C22—H22	120.7
O1W—Co1—O5^i^	90.33 (9)	C23—C22—H22	120.7
O2—Co1—O6^i^	89.58 (8)	N2—C23—C22	123.0 (3)
N2—Co1—O6^i^	150.47 (9)	N2—C23—C24	114.6 (2)
N1—Co1—O6^i^	99.27 (9)	C22—C23—C24	122.4 (3)
O1W—Co1—O6^i^	89.73 (8)	N1—C24—C25	122.7 (3)
O5^i^—Co1—O6^i^	59.93 (8)	N1—C24—C23	114.4 (2)
O12—Co2—N3	119.99 (9)	C25—C24—C23	122.9 (3)
O12—Co2—N4	92.54 (9)	C26—C25—C24	117.9 (3)
N3—Co2—N4	77.48 (10)	C26—C25—H25	121.0
O12—Co2—O2W	86.76 (9)	C24—C25—H25	121.0
N3—Co2—O2W	95.71 (9)	C25—C26—C27	119.2 (3)
N4—Co2—O2W	171.71 (10)	C25—C26—H26	120.4
O12—Co2—O10^ii^	149.51 (9)	C27—C26—H26	120.4
N3—Co2—O10^ii^	90.50 (9)	C28—C27—C26	120.0 (3)
N4—Co2—O10^ii^	94.22 (9)	C28—C27—H27	120.0
O2W—Co2—O10^ii^	90.54 (9)	C26—C27—H27	120.0
O12—Co2—O9^ii^	90.11 (8)	N1—C28—C27	121.8 (3)
N3—Co2—O9^ii^	149.55 (8)	N1—C28—H28	119.1
N4—Co2—O9^ii^	98.13 (9)	C27—C28—H28	119.1
O2W—Co2—O9^ii^	90.14 (8)	O1—C29—O2	124.4 (3)
O10^ii^—Co2—O9^ii^	59.50 (8)	O1—C29—C30	119.5 (3)
N3—C1—C2	122.0 (4)	O2—C29—C30	116.0 (3)
N3—C1—H1	119.0	C32—C30—C31	119.6 (2)
C2—C1—H1	119.0	C32—C30—C29	118.4 (3)
C3—C2—C1	120.1 (4)	C31—C30—C29	121.9 (2)
C3—C2—H2	120.0	C33—C31—C30	118.9 (3)
C1—C2—H2	120.0	C33—C31—H31	120.6
C4—C3—C2	118.6 (3)	C30—C31—H31	120.6
C4—C3—H3	120.7	C30—C32—C34	120.3 (3)
C2—C3—H3	120.7	C30—C32—H32	119.9
C3—C4—C5	118.8 (3)	C34—C32—H32	119.9
C3—C4—H4	120.6	C35—C33—C31	122.8 (3)
C5—C4—H4	120.6	C35—C33—N6	118.6 (3)
N3—C5—C4	122.7 (3)	C31—C33—N6	118.5 (3)
N3—C5—C6	113.9 (3)	C32—C34—C35	120.5 (3)
C4—C5—C6	123.4 (3)	C32—C34—C36	119.2 (3)
N4—C6—C7	121.6 (3)	C35—C34—C36	120.2 (2)
N4—C6—C5	115.2 (3)	C33—C35—C34	117.9 (3)
C7—C6—C5	123.2 (3)	C33—C35—H35	121.0
C8—C7—C6	118.2 (3)	C34—C35—H35	121.0
C8—C7—H7	120.9	O6—C36—O5	121.3 (3)
C6—C7—H7	120.9	O6—C36—C34	119.4 (3)
C7—C8—C9	119.5 (3)	O5—C36—C34	119.3 (3)
C7—C8—H8	120.2	O6—C36—Co1^ii^	63.61 (16)
C9—C8—H8	120.3	O5—C36—Co1^ii^	57.85 (15)
C10—C9—C8	120.0 (4)	C34—C36—Co1^ii^	174.8 (2)
C10—C9—H9	120.0	C28—N1—C24	118.4 (3)
C8—C9—H9	120.0	C28—N1—Co1	125.6 (2)
N4—C10—C9	121.6 (3)	C24—N1—Co1	115.95 (19)
N4—C10—H10	119.2	C19—N2—C23	118.0 (3)
C9—C10—H10	119.2	C19—N2—Co1	124.5 (2)
C12—C11—C17	119.6 (3)	C23—N2—Co1	117.12 (19)
C12—C11—H11	120.2	C1—N3—C5	117.8 (3)
C17—C11—H11	120.2	C1—N3—Co2	124.4 (2)
C13—C12—C11	122.3 (3)	C5—N3—Co2	117.2 (2)
C13—C12—N5	118.7 (3)	C10—N4—C6	119.1 (3)
C11—C12—N5	119.0 (3)	C10—N4—Co2	125.1 (2)
C12—C13—C14	118.0 (3)	C6—N4—Co2	115.9 (2)
C12—C13—H13	121.0	O7—N5—O8	122.6 (3)
C14—C13—H13	121.0	O7—N5—C12	118.7 (3)
C16—C14—C13	120.3 (3)	O8—N5—C12	118.7 (3)
C16—C14—C15	119.0 (3)	O3—N6—O4	122.7 (3)
C13—C14—C15	120.7 (2)	O3—N6—C33	119.3 (3)
O9—C15—O10	121.7 (3)	O4—N6—C33	118.0 (3)
O9—C15—C14	119.4 (3)	C29—O2—Co1	120.23 (19)
O10—C15—C14	118.9 (2)	C36—O5—Co1^ii^	92.08 (17)
C17—C16—C14	120.8 (3)	C36—O6—Co1^ii^	86.49 (18)
C17—C16—H16	119.6	C15—O9—Co2^i^	85.29 (18)
C14—C16—H16	119.6	C15—O10—Co2^i^	93.31 (17)
C16—C17—C11	119.0 (3)	C18—O12—Co2	121.93 (19)
C16—C17—C18	118.5 (3)	Co1—O1W—H1W	105 (3)
C11—C17—C18	122.5 (3)	Co1—O1W—H2W	115 (3)
O11—C18—O12	124.9 (3)	H1W—O1W—H2W	111.4 (18)
O11—C18—C17	120.0 (3)	Co2—O2W—H3W	111 (3)
O12—C18—C17	115.1 (3)	Co2—O2W—H4W	114 (3)
N2—C19—C20	121.7 (3)	H3W—O2W—H4W	111.0 (17)
N2—C19—H19	119.1		

Symmetry codes: (i) *x*+1, *y*, *z*; (ii) *x*−1, *y*, *z*.

RETRACTED

### Hydrogen-bond geometry (Å, °)

**Table:**

*D*—H···*A*	*D*—H	H···*A*	*D*···*A*	*D*—H···*A*
O1W—H1W···O12^i^	0.830 (10)	2.01 (2)	2.771 (3)	153 (3)
O2W—H4W···O2^ii^	0.831 (10)	1.957 (17)	2.747 (3)	159 (3)
O1W—H2W···O9	0.830 (10)	2.05 (2)	2.763 (3)	143 (3)
O2W—H3W···O6	0.835 (10)	2.10 (3)	2.781 (3)	138 (3)

Symmetry codes: (i) *x*+1, *y*, *z*; (ii) *x*−1, *y*, *z*.
